# Current Status of Fear of Disease Progression in Patients with Advanced Cancer and Usefulness of Dignity Therapy Intervention

**DOI:** 10.1155/2022/6069060

**Published:** 2022-03-21

**Authors:** Yongli Zhang, Fangru Zhou, Hong Yang, Xue Gong, Jingfang Gao

**Affiliations:** ^1^Department of Hematology, Shijiazhuang People's Hospital, Shijiazhuang 050000, China; ^2^Department of Oncology, Shijiazhuang First Hospital, Shijiazhuang 050000, China

## Abstract

With changes in lifestyle and an increase in bad health habits, cancer has become a noncommunicable and frequently occurring disease that poses a serious threat to human life. *Cancer* is associated with high rates of morbidity and mortality worldwide. As a major negative life event, advanced malignancies lead to strong mood swings in most patients. Furthermore, various internal and external factors can have a huge impact on patients' physical and mental health and put them in a stressful situation, causing a series of psychological stress responses. To explore the degree of fear of disease progression in patients with advanced cancer and the usefulness of dignity therapy. Overall, 120 patients with advanced malignant tumors admitted to Shijiazhuang No. 1 hospital between January 2019 and January 2020 were enrolled. The selected patients were divided into the test and control groups (60 people per group) using a random number table. All patients received basic treatment. Patients in the trial group also received dignity therapy. The intervention period was 4 weeks. Simplified scales were used for assessing disease progression (FoP-Q-SF) and quality of life (QLQ-C30) before and after the intervention, and the scores were compared between the groups. After the intervention, the degree of fear in the experimental group was lower than that of the control group. Cognitive function, emotional function, and the scores of the overall health status of the experimental group were higher than those of the control group. Additionally, the scores of fatigue, insomnia, loss of appetite, and diarrhea in the experimental group were lower than those of the control group (*P* < 0.05). The social support level scale scores, depression scores, hospital anxiety and depression scale scores, and patient dignity inventory scores of the experimental group were lower than those of the control group (*P* < 0.05). Patients with advanced malignant tumors have fear, anxiety, and depression related to disease progression. Dignity therapy is useful for improving the patients' quality of life, increasing dignity, and enhancing social support.

## 1. Introduction

Negative mood, including anxiety and fear, can cause cognitive and behavioral changes in patients, which manifest as self-criticism, self-efficacy, self-esteem, avoidance, and other nonadaptive behaviors, resulting in varying degrees of decline in quality of life [1–3]. With the development of modern medical models, dignity therapy, which is based on empirical individualized psychological intervention treatment, can help clinicians in maintaining the patients' dignity and decreasing psychological pain in the terminal stage through simple interviews. This provides opportunities for patients to open up and express their inner feelings, to review what is the most meaningful and valuable to them at the end of life to encourage patients to regain confidence, and to feel the care from family and society, and, consequently, to increase their will to live [4, 5]. Currently, dignity therapy is started late in Chinese patients with advanced cancer. Our paper analyzed the degree of fear of disease progression in patients with advanced malignant tumors and the clinical value of dignity therapy intervention.

The rest of this paper is organized as follows: section 2 discusses materials and methods. Comparison of experimental results between the two groups is discussed in section 3.  Section 4 shows the experimental results analysis, and section 5 concludes the paper with a summary and future research directions.

## 2. Materials and Methods

### 2.1. Data

Overall, 120 patients with advanced malignant tumors admitted to Shijiazhuang No. 1 hospital between January 2019 and January 2020 were selected as research subjects. The patients included in the paper were divided into the experimental group (cases) and the control group by a random number table, with 60 patients in each group. The inclusion criteria were as follows: (1) patients' age ranged from 45 to 79 years old; (2) patients were pathologically confirmed to have an advanced malignant tumor (TNM stage ≥ III); (3) the patient was conscious, received treatment in the oncology department of our hospital, and had a normal level of language and communication ability; and (4) the survival time was estimated to be no less than three months. The exclusion criteria were as follows: (1) patients with major diseases of other body systems (severe cerebrovascular diseases, acute myocardial infarction, severe heart failure, etc.), (2) patients who were able to live independently, (3) patients with senile dementia and mental diseases, and (4) patients with other serious diseases affecting the quality of life.

Before paper initiation, the paper plan was submitted to the Medical Ethics Committee of Shijiazhuang First Hospital for approval, and the paper was conducted after the medical ethics committee made a decision and published a document (Document No. Hospital (London) Office ([2018] No. 24). The paper protocol provided informed consent from patients and their families.

### 2.2. Basic Treatment

Reasonable radiotherapy, chemotherapy, and molecular targeted therapy were selected according to the development and characteristics of patients with tumors. Dynamic observation of disease changes was carried out after the improvement of relevant examinations. Patients were given psychological counseling, support, and encouragement, which helped them build confidence and have an optimistic attitude to face treatment. Discharge guidance was provided, and patients were instructed to live routinely to ensure adequate rest, and a review was performed when necessary.

### 2.3. Dignity Therapy

A dignity therapy intervention team was established, including three specialists, one dignity therapy expert, and six responsible nurses. The dignity therapy experts were responsible for the guidance of dignity overall care. An oncologist was responsible for disease assessment and staging diagnosis, and the nurse was responsible for dignity interview introduction, appointment, recording, and conversion. Special training for personnel was carried out, and 12-hour training and assessment of the implementation content, research purpose, significance, dignity interview skills and precautions, recording conversion, editing, sorting, and so on. The interview outline of dignity was determined, including important memories of patients, about themselves, life roles, personal achievements, specific things, expectations and wishes, experiences, and instructions. A dignity therapy brochure was prepared by the team, which mainly included the definition of dignity therapy, core purpose, applicable group, people who should implement it, interview method, interview time, interview place, interview content, inheritance document, and inheritance. The brochures were distributed by the responsible nurse to patients and their families when patients were admitted to the hospital, and they were also instructed to read them to better help patients and their families know and understand dignity therapy. After the patient was admitted to the hospital, the responsible nurse introduced dignity therapy, made an interview appointment with the patient, and completed the collection of patient data. A formal dignity interview was conducted according to the scheduled interview time; the number of interviews was 1-2, and the interview time was no more than 60 min per interview. After communicating with the patient and confirming the interview time and place again, the interviewee arranged an interview room that was clean, warm, and comfortable 1 h before the interview, prepared fresh fruit, candy, and tissues, and adjusted the recording equipment. Dignity therapy was introduced again, and patients talked one by one according to the order of the dignity interview outline. In the interview process, patients were actively listened to and appropriately guided, and they controlled the interview time well so as to help them with psychological relief from emotional breakdown when talking about important experiences in the interview process, and at the same time, they were given spiritual care and encouragement. The narrative text was returned to the patient within five working days after the interview; within 2 days after the dignity interview, the interviewer completed the recording conversion. After printing the original text, the expert accompanied the patient to carefully read and check the contents that the patient decided to retain, adjust, and delete with different colors. On the third day after the interview, the document was edited according to the marked original text. After printing, the document was checked with the patient again, and the revised text was prepared on the same day as required by the patient. The revised text had to be printed, bound, and returned to the patient within the specified time, and the patient should be informed of the right to choose whom to share the document with or with whom to pass it on.

### 2.4. Evaluation Scale and Its Methods

The simplified disease progression scale (FOP-Q-SF) [6] score, quality of life (QLQ-C30) score, social support scale (SSRS) [7, 8], hospital anxiety and depression scale (HADS) [9] score, and patient dignity inventory (PDI) [10] scores were compared between the two groups before and after the intervention.

The simplified disease progression scale (FOP-Q-SF) contains a total of 12 questionnaire items, and the Likert 5-level scoring method was used for each item. The total score ranges from 12 to 60, with a total score of >20 indicating mild fear, a total score of >32 indicating moderate fear, and a total score of >39 indicating severe fear.

A quality of life (QLQ-C30) score was used to measure the quality of life of patients with cancer, including functional dimensions, symptom dimensions, and overall health dimensions. The higher the scores of functional dimensions and overall health dimensions, the better the quality of life of patients. The higher the symptom dimension score, the more severe the patients' symptoms are.

The social support scale (SSRS) was developed by Xiao Shuiyuan and was mainly evaluated in three aspects: objective support, subjective support, and utilization of support. The total SSRS score was 66 points, and the higher the total score, the higher the social support of patients.

The hospital anxiety depression scale (HADS) contains the following items: “I feel nervous or excited,” “I am still interested in things that I was interested in the past,” “I was afraid, and it seems to be a serious matter to occur.” There are 14 questionnaire items, including seven questions for the anxiety score, and the other seven related to the depression score, including anxiety and depression. These are part of the total score of 0–21 points, and a score above 8 is considered to indicate anxiety or depression.

The dignity scale (PDI) was revised by Cao Yanmei et al., with 25 items and five dimensions. A Likert level 5 scoring method was used for each item. The total score was 25–125.

### 2.5. Statistical Analysis

Data of body mass index (BMI) and years of education of patients in this paper had approximate normal distribution or normal distribution by normal distribution test, represented by ($\bar{x}$ ± *s*). Comparisons between groups were compared using the *t*-test. The enumeration data were expressed as percentages, and the *χ*^2^ test was used for comparison. The professional SPSS software (version 21.0) was used for data processing, and the test level was *α* = 0.05.

## 3. Results

### 3.1. Comparison of Baseline Data between the Two Groups

There was no significant difference in baseline data, including age, BMI, years of education, sex, and marriage, between the experimental group and the control group (*P* > 0.05).  Table 1 is a comparison of baseline data between the two groups.

### 3.2. Comparison of the Degree of Fear of Disease between the Two Groups

Before the intervention, there was no significant difference in the degree of fear of disease between the experimental group and the control group (*P* > 0.05).  Table 2 shows a comparison of the degree of fear between the two groups before the intervention.

After the intervention, the degree of fear of disease in the experimental group was lower than that of the control group, and the difference was significant (*P* < 0.05).  Table 3 presents a comparison of the degree of fear between the two groups after the intervention.

### 3.3. Comparison of Quality of Life Scores between the Two Groups before and after the Intervention

Before the intervention, the experimental group and the control group had no significant differences in the functional dimensions, symptom dimensions, and overall health dimension scores (*P* > 0.05). After the intervention, the experimental group's role function, cognitive function, emotional function, and the scores of overall health status were higher than those of the control group (*P* < 0.05), and the scores of fatigue, insomnia, loss of appetite, and diarrhea in the test group were lower than those of the control group (*P* < 0.05).  Table 4 is a comparison of quality-of-life scores between the two groups before and after the intervention.

### 3.4. Comparison of Social Support Level Scale Scores between the Two Groups before and after the Intervention

Before the intervention, there were no significant differences in objective support, subjective support, utilization of support, and social support level scale scores between the experimental group and the control group (*P* > 0.05). After the intervention, the social support level scale scores of the experimental group were lower than those of the control group (*P* < 0.05).  Table 5 displays a comparison of social support level scale scores between the two groups before and after the intervention.

### 3.5. Comparison of HADS Scores between the Two Groups before and after the Intervention

Before the intervention, the HADS scores of the experimental group and the control group were not significantly different (*P* > 0.05). After the intervention, the depression and HADS scores of the experimental group were lower than those of the control group (*P* < 0.05).  Table 6 shows a comparison of HADS scores between the two groups before and after the intervention.

### 3.6. Comparison of PDI Scores between the Two Groups before and after the Intervention

Before the intervention, the PDI scores of the experimental group and the control group did not show any significant difference (*P* > 0.05). After the intervention, the PDI scores of the experimental group were lower than those of the control group (*P* < 0.05).  Table 7 is a comparison of PDI scores between the two groups before and after the intervention.

## 4. Experimental Results Analysis

In this paper, the role function, cognitive function, emotional function, and overall health score of the experimental group were higher than those of the control group after the intervention. After the intervention, the scores of fatigue, insomnia, loss of appetite, and diarrhea in the experimental group were lower than those of the control group, suggesting that dignity therapy intervention can effectively improve the quality of life of patients with advanced cancer.

In recent years, with changes in the modern medical model, there has been a shift from simply maintaining patients' lives and organ functions to improving their quality of life [11, 12]. The traditional functional system of nursing mode pays attention to the physical rehabilitation of the patients but ignores the adjustment of their psychological states, and the functional system of nursing mode can lead to a mindset in medical nursing staff. Nurses focus only on the execution of medical orders and therapeutic nursing operations; they do not often pay attention to the content of nursing services.

Based on empirical individualized psychological intervention treatment, dignity therapy has been applied to patients with advanced cancer, which must be performed by medical personnel trained in dignity therapy [13, 14]. A problem outline with dignity therapy was adopted, and the form of semistructured interview recording for patients with the end-stage disease can provide opportunities to talk about important life experiences and share feelings and emotions [15]. The interview recording was transformed into a narrative text for the patient and family to save and inherit, and patients were allowed to share information with the person they love so as to make the patient's personal value persist beyond their own death, help them alleviate psychological pain, and regain the value of life meaning so that they spend the last years of life with dignity [15].

Quality of life is a comprehensive evaluation of the good adaptation in physical, psychological, and social function that an individual or a group feels about, which focuses more on the patient's subjective feelings and functions and is a multidimensional evaluation index of the individual or group's health. Patients with cancer can experience pain, insomnia, loss of appetite, and body function; there will also be pessimism, depression, hopelessness, meaninglessness, and other psychological and mental state changes, and the overall quality of life and its dimensions are generally low [16, 17]. The application of dignity therapy can effectively improve emotional and social functions in patients with advanced cancer, which is beneficial for promoting positive emotions toward life events and helping them integrate better into family life and social activities, making it easier to express real inner feelings to achieve a more peaceful state of mood [18].

In this paper, the degree of fear in the experimental group was lower than that of the control group after the intervention, suggesting that dignity therapy can effectively reduce the psychological state of fear in patients with advanced cancer. After the intervention, the social support scale score of the experimental group was lower than that of the control group, suggesting that the dignity therapy intervention for patients with advanced cancer is helpful for improving the degree of social support for patients. Dignity therapy can provide opportunities for patients with advanced cancer to express real feelings, reinterpret the meaning of their life, and recall what is most valuable and meaningful to them and the spiritual wealth they want to leave to their loved ones and friends, enhancing their sense of value and dignity, so that they can regain their enthusiasm for life at this stage of illness. Patients in the process of constantly recalling the valuable and meaningful past can enhance their sense of self-worth and significance, and they can be encouraged to express ideas to share with relatives and friends, learn to be relieved, and gradually obtain inner peace [19].

In addition, the paper also suggests that dignity therapy intervention for patients with advanced cancer is helpful for improving patients' dignity. When the individual lives of patients with advanced malignant tumor face a threat, a review of the past events can occur naturally and instinctively. Regardless of the positive or negative events of the past, patients would want to recall and share with their loved ones, especially summed up from feelings and experience. If the demand can be realized, then patients can gain a more positive attitude, establish a closer relationship with their relatives, enhance their confidence in the face of disease, improve their hope level, and change their negative emotions [20]. This paper analyzed the common psychological burden of fear and negative emotions in patients with advanced cancer. The dignity of patients is closely related to their quality of life. Dignity therapy can provide psychological support and counseling for patients and explore their inner sense of self-worth and dignity. The improvement in the sense of dignity of patients with advanced cancer through preliminary attention and in-depth discussion is still the focus of future research in the field of clinical care for patients with cancer.

## 5. Conclusion

In conclusion, patients with advanced malignant tumor diseases have fear, anxiety, and depression related to disease progression. The use of dignity therapy intervention has a certain value in improving the quality of life of patients, increasing their sense of dignity, and enhancing their sense of social support.

This paper has some limitations, which should be considered. In this paper, objective indicators were not included, and their effect after the intervention was not evaluated because of the disunity of disease diagnosis and the complex and unstable condition of patients with advanced cancer. Our findings suggest that, in the future, targeted intervention should be provided to patients according to the type of cancer, and objective indicators corresponding to the disease should be adopted to evaluate the outcome. In addition, the narrative text formed by the dignity interview in the paper was returned only to the patients and their families in the form of documents, in a slightly monotonous form. In the future, more information about patients can be collected according to their content to help patients save more meaningful and valuable memories.

## Figures and Tables

**Table 1:** Comparison of baseline data between the two groups.

Groups	Experimental group (*n* = 60)	Control group (*n* = 60)	t/*χ*^2^ value	*P* value
Age (years old)	56.9 ± 6.3	58.0 ± 6.0	−0.979	0.329
BMI (kg/m^2^)	22.5 ± 2.0	22.2 ± 2.4	0.744	0.458
Education year (years)	8.9 ± 2.2	8.5 ± 2.4	0.952	0.343
Gender (%)			1.250	0.264
Male	39 (65.00)	33 (55.00)		
Female	21 (35.00)	27 (45.00)		
Marriage (%)			2.163	0.339
Married	51 (85.00)	54 (90.00)		
Unmarried	2 (3.33)	0 (0.00)		
Widowed/divorced	7 (11.67)	6 (10.00)		
Major caregiver (%)			2.063	0.356
Spouse	45 (75.00)	38 (63.33)		
Offspring	13 (21.67)	18 (30.00)		
Others	2 (3.33)	4 (6.67)		
Family monthly income			2.823	0.244
＜3000 yuan	11 (18.33)	7 (11.67)		
3000～6000 yuan	34 (56.67)	30 (50.00)		
≥6000 yuan	15 (25.00)	23 (38.33)		
Pay way (%)			1.681	0.432
Urban and rural residents	24 (40.00)	28 (46.67)		
Town workers	36 (60.00)	31 (51.67)		
Self-paying	0 (0.00)	1 (1.67)		
Cancer type (%)			1.414	0.702
Lung cancer	21 (35.00)	18 (30.00)		
Colorectal cancer	18 (30.00)	24 (40.00)		
Liver cancer	8 (13.33)	6 (10.00)		
Others	13 (21.67)	12 (20.00)		
TNM staging (%)			1.319	0.251
Stage III	36 (60.00)	42 (70.00)		
Stage IV	24 (40.00)	18 (30.00)		

**Table 2:** Comparison of the degree of fear between the two groups before the intervention [*n* (%)].

Groups	*n*	No fear	Mild fear	Moderate fear	Severe fear
Experimental group	60	6 (10.00)	15 (25.00)	24 (40.00)	15 (25.00)
Control group	60	3 (5.00)	11 (18.33)	34 (56.67)	12 (20.00)
Z value		−0.618			
*P* Value		0.537			

**Table 3:** Comparison of the degree of fear between the two groups after the intervention [*n* (%)].

Groups	*n*	No fear	Mild fear	Moderate fear	Severe fear
Experimental group	60	11 (18.33)	39 (65)	8 (13.33)	2 (3.33)
Control group	60	8 (13.33)	30 (50)	17 (28.33)	5 (8.33)
*Z* value		−2.187			
*P* Value		0.029			

**Table 4:** Comparison of quality-of-life scores between the two groups before and after the intervention ($\bar{x}$ ± *s*, points).

Items	Before intervention		*T* value	*P* value	After intervention		*T* value	*P* value
	Experimental group (*n* = 60)	Control group (*n* = 60)			Experimental group (*n* = 60)	Control group (*n* = 60)		
*Functional dimensions*								
Symptom dimensions	8.53 ± 1.77	8.76 ± 1.80	−0.706	0.482	8.80 ± 2.03	8.38 ± 2.24	1.076	0.284
Role function	2.30 ± 0.84	2.41 ± 0.79	−0.739	0.461	3.25 ± 0.78	2.75 ± 0.71	3.672	0.000
Cognitive function	3.68 ± 0.94	3.80 ± 0.98	−0.685	0.495	4.61 ± 1.05	4.13 ± 0.96	2.613	0.010
Emotional function	6.84 ± 1.32	6.73 ± 1.18	0.481	0.631	8.25 ± 1.50	7.10 ± 1.48	4.227	0.000
Social function	3.63 ± 0.86	3.81 ± 0.92	−1.107	0.270	3.81 ± 0.95	3.66 ± 0.85	0.911	0.364
Overall health status	7.74 ± 1.22	7.98 ± 1.13	−1.118	0.266	8.68 ± 1.30	7.88 ± 1.36	3.294	0.001
*Functional dimensions*								
Fatigue	2.85 ± 0.64	2.93 ± 0.62	−0.695	0.488	1.84 ± 0.55	2.54 ± 0.61	-6.602	0.000
Insomnia	2.73 ± 0.61	2.85 ± 0.59	−1.095	0.276	2.60 ± 0.66	2.71 ± 0.56	-0.984	0.327
Nausea and vomiting	2.24 ± 0.58	2.40 ± 0.65	−1.423	0.157	2.18 ± 0.56	2.32 ± 0.60	−1.321	0.189
Dyspnea	1.84 ± 0.44	1.77 ± 0.42	0.891	0.375	1.77 ± 0.48	1.85 ± 0.43	−0.962	0.338
Insomnia	2.21 ± 0.57	2.12 ± 0.51	0.911	0.364	1.48 ± 0.30	1.87 ± 0.48	−5.337	0.000
Loss of appetite	2.36 ± 0.55	2.24 ± 0.57	1.174	0.243	1.55 ± 0.42	2.16 ± 0.51	−7.152	0.000
Astriction	1.94 ± 0.42	1.86 ± 0.40	1.068	0.288	1.88 ± 0.38	1.98 ± 0.40	−1.404	0.163
Diarrhea	2.06 ± 0.47	2.12 ± 0.43	-0.730	0.467	1.72 ± 0.40	2.01 ± 0.48	−3.595	0.000
Economic difficulty	2.95 ± 0.73	3.10 ± 0.81	−1.066	0.289	3.05 ± 0.78	3.16 ± 0.83	−0.748	0.456

**Table 5:** Comparison of social support level scale scores between the two groups before and after the intervention ($\bar{x}$ ± *s*, points).

Groups	N	Before intervention	After intervention	Before intervention	After intervention
		Objective support		Subjective support	

Experimental group	60	8.75 ± 2.80	12.28 ± 3.16	19.64 ± 3.84	24.63 ± 4.36
Control group	60	9.10 ± 2.55	10.45 ± 3.32	20.71 ± 4.02	22.28 ± 4.51
*t* value		−0.716	3.093	−1.491	2.902
*P* value		0.475	0.002	0.139	0.004
		Utilization of support		Total score	
Experimental group	60	5.52 ± 1.47	7.10 ± 1.94	33.91 ± 6.83	44.01 ± 7.54
Control group	60	5.83 ± 1.62	6.29 ± 2.00	35.64 ± 6.90	39.02 ± 7.76
*T* value		−1.098	2.252	−1.380	3.572
*P* value		0.275	0.026	0.170	0.001

**Table 6:** Comparison of HADS scores between the two groups before and after the intervention ($\bar{x}$ ± *s*, points).

Groups	*N*	Anxiety scores		Depression scores		HADS	
		Before intervention	After intervention	Before intervention	After intervention	Before intervention	After intervention
Experimental group	60	13.84 ± 2.82	10.59 ± 2.87	14.26 ± 3.11	8.84 ± 2.51	28.10 ± 4.62	19.43 ± 3.95
Control group	60	13.51 ± 2.93	11.25 ± 2.73	13.81 ± 3.34	10.74 ± 2.84	27.32 ± 4.18	21.99 ± 4.20
*T* value		0.629	−1.291	0.764	−3.883	0.970	−3.439
*P* value		0.531	0.199	0.447	0.000	0.334	0.001

HADS, hospital anxiety and depression scale.

**Table 7:** Comparison of PDI scores between the two groups before and after the intervention ($\bar{x}$ ± *s*, points).

Groups	N	PDI scores		*T* value	*P* value
		Before intervention	After intervention		
Experimental group	60	54.86 ± 11.20	23.74 ± 5.11	19.581	0.000
Control group	60	56.92 ± 12.42	27.83 ± 6.35	16.154	0.000
t value		-0.954	-3.887		
*P* Value		0.342	0.000		

PDI, patient dignity inventory.

## Data Availability

The data used to support the findings of this paper are available from the author upon request.
